# A Variable-Clustering-Based Feature Selection to Improve Positive and Negative Discrimination of P53 Protein in Colorectal Cancer Patients

**DOI:** 10.1155/2022/9261713

**Published:** 2022-11-17

**Authors:** Luqing Wang, Li Feng, Jiasi Wang, Jie Li, Hongbin Li, Fanxin Zeng, Liangli Sun

**Affiliations:** ^1^Faculty of Innovation Engineering, Macau University of Science & Technology, Macau, China; ^2^Department of Clinical Laboratory, Dazhou Central Hospital, Dazhou, Sichuan, China; ^3^Department of Clinical Research Center, Dazhou Central Hospital, Dazhou, Sichuan, China; ^4^Department of Respiratory Medicine, Dazhou Central Hospital, Dazhou, Sichuan, China; ^5^Department of Rheumatology and Immunology, Dazhou Central Hospital, Dazhou, Sichuan, China

## Abstract

P53 protein tumor suppressor gene plays a guiding role in the treatment and prognosis of colorectal cancer (CRC). This paper aimed at proposing a feature selection method based on variable clustering to improve positive and negative discrimination of P53 protein in CRC patients. In this approach, we cluster the preprocessed dataset with variables, and then find the features with the largest information value (IV) for each cluster to form a feature subset. We call this method as IV_Cluster. In the actual medical data test, compared with the information value feature selection method, the accuracy of the 10-fold cross-validation logistic regression model increased by 4.4%, 2.0%, and 5.8%, and Kappa values increased by 21.8%, 8.6%, and 22.4%, respectively, under 5, 10, and 15 feature sets.

## 1. Introduction

Feature selection method is a data preprocessing approach that selects feature subspaces from the original feature space that contribute to the target [1–3]. Feature selection methods have been studied and applied in clinical and even imaging studies. Feature selection method is an effective means to deal with small sample high-dimensional data. According to whether the processed dataset has labels, it can be divided into supervised feature selection and unsupervised feature selection. The former is to select a series of feature sets that are effective for labels; the latter is used to select features that can maintain the feature structure and achieve reduction. According to the strategy of feature selection, it can be divided into filtering, wrapping, and embedding. Filtering is a selection method based on feature scoring, which is simple and efficient, and is often used for processing high-dimensional data. Wrapping is a method that evaluates selected subsets based on a black-box model to select the best subset. It takes into account the interaction between features, which takes a long time and computation. Embedding is a method to measure the importance of features in the construction of the model. However, there are many current feature selection methods. How to select and design a suitable feature selection algorithm is a confusing and even difficult thing for clinical medical research.

Variable clustering is a kind of unsupervised learning paradigm of variable structure to achieve the goal of dimensionality reduction. Variable clustering has also been widely studied and applied in feature selection. For example, variable clustering based on K-means [4], a fast hybrid feature selection based on correlation-guided clustering and particle swarm optimization for high-dimensional data [5], clustering-guided particle swarm feature selection algorithm for high-dimensional imbalanced data with missing values [6].

We collected a medical dataset of P53 protein in colorectal cancer (CRC), which included imaging features, other clinical features, and serum tumor marker features, as well as P53 protein negative and positive features. Our goal was to investigate the relationship between these feature sets and the negative and positive expressions of P53 protein. The P53 protein encoded by wild-type TP53 gene is maintained at a low level in normal cells and regulates gene transcription to respond to adverse factors such as oncogene signal activation and DNA damage. When TP53 gene is mutated, the P53 protein encoded by TP53 gene has a long half-life and strong stability, which can accumulate continuously in the nucleus and lose its monitoring effect on cells. On the contrary, it acts as an oncogene in cell malignancy, promoting invasion, metastasis, proliferation, and cell survival.

After TP53 mutation occurs in CRC patients, 50% to 75% of the cases are positive [7]. P53 mutations are associated with lymphatic infiltration in proximal colon cancer, and are significantly associated with lymphatic and vascular infiltration in distal CRC. Compared with P53 wild-type, patients with P53 mutant CRC have higher degree of chemotherapy resistance and poorer prognosis [8, 9]. In recent years, it has been found that P53 protein expression is significantly correlated with TP53 gene status [10]. Therefore, immunohistochemical method is commonly used to detect P53 protein expression to reflect TP53 gene mutation status in clinical practice. Imaging omics is an emerging quantitative analysis method based on high throughput characteristics of medical images. More and more evidences show that as a noninvasive method, it has advantages in early diagnosis, prognosis prediction, and efficacy evaluation of tumors [11–15]. Chen et al. found that texture features extracted by PET/CT can provide supplementary information for the determination of TP53 gene changes in CRC [16]. Although there is little evidence to support a direct correlation between texture heterogeneity and any specific underlying physiological process or biological heterogeneity, a large number of current studies suggest that there is a correlation between imaging phenotypes and mutant landscapes, gene expression, and signaling pathways [17]. At present, there are very few articles about the relationship between P53 and other clinical features such as imaging, and our practice shows that the effect of common feature selection methods is not ideal. We expect further improvement.

This work provides a variable clustering based feature selection to improve positive and negative discrimination of P53 protein in CRC patients. The similarity of variables is described by an unsupervised learning method (K-means), in which a series of target groups are divided, and the feature that maximizes the variable information value (IV) is selected as a representative from each group, thereby forming a new feature subset, and this method is recorded as IV_Cluster. The following are the three primary contributions of this paper:

1. Develop a variable clustering IV feature selection approach that incorporates unsupervised and supervised learning concepts
2. The actual clinical colon cancer tumor medical dataset used to pick features by this method
3. The capacity to distinguish between the negative and positive forms of the P53 protein has improved as a result of this feature selection

This paper is organized as follows: the introduction is done in Section 1.  Section 2 describes the relevant knowledge then the detailed introduction of the variable clustering IV feature selection algorithm is done Section 3. The experimental results and analysis is illustrated in Section 4. The discussion is shown in Section 5, while Section 6 contains the conclusion.

## 2. Prerequisites

The relevant knowledge in the paper includes variable binning, data WOE encoding, information value definition, and an introduction to the logistic regression algorithm.

### 2.1. Variable Binning

In this paper, we apply an optimal variable partitioning technique, which is a conditional inference tree [18–20]. It belongs to a supervised variable sorting technology, which realizes an unbiased variable sorting technology by means of recursion and statistical hypothesis testing.

### 2.2. Weight of Evidence (WOE) Encoding

After the variable binning of the dataset, we can perform weight of evidence (WOE) coding on the binning of each variable [20–23]. The calculation formula of WOE is

(1) $$\begin{array}{c} \text{WOE}\left(x\right)=\log\left(\frac{f\left(x\left|y=1\right.\right)}{f\left(x\left|y=0\right.\right)}\right). \end{array}$$

The denominator and numerator in this formula represent the proportion of negative and positive in the subset of each variable bin, respectively. Variable WOE encoding makes the data more robust and improves the interpretability of the results.

### 2.3. Information Value (IV) of Variable

The IV of the variable [20, 22] is used to describe the discriminative ability of the variable to the target variable. Calculated as follows:

(2) $$\begin{array}{c} IV=\underset{x}{\sum }\left(f\left(\left.x\right|1\right)-f\left(\left.x\right|0\right)\right)\text{WOE}\left(x\right). \end{array}$$

Variable IV is a filtered feature selection that has the advantage of being simple and effective. We can use Top-K or Top-Percentage strategies to select variables based on their IV values. This paper adopts the Top-K strategy for testing and verification.

### 2.4. Logistical Regression Model

The logistic regression model [24–26] is a classic binary classification model that is simple and easy to interpret. LR model is mathematically equivalent to solving an unconstrained optimization problem, the formula is as follows:

(3) $$\begin{array}{c} \underset{\begin{array}{c} w\in R^{k}\\ b\in R \end{array}}{\min}\frac{1}{N}\overset{N}{\underset{i=1}{\sum }}\log\left(1+e^{\left[-y_{i}\left(w^{T}x_{i}+b\right)\right]}\right). \end{array}$$

## 3. Materials and Methods

This work proposes an IV_Cluster feature selection method. This method includes three important steps. We use the conditional inference tree to optimally bin the variables and calculate the IV value of the variable, and then perform cluster learning on the variables and select the feature with the largest IV value in each cluster. A logistic regression model with 10 cross-validations was performed on a good feature set and the performance differences of all features and IV selected features were compared and analyzed.

### 3.1. Datasets

This proposed method is designed to process a small sample high-dimensional dataset of the P53 proteome of colorectal cancer. This dataset is derived from the image dataset of Dazhou Central People's Hospital in Sichuan Province, and obtained a dataset of 349 patients and 867 features. These features include the basic information of patients, laboratory information, and imaging-based wavelet features to extract P53 protein group information.

#### 3.1.1. Data Preprocessing

*(1) Missing Value Processing*. For the dataset, first do the missing detection, and then use the following method to process the features with missing values. The numerical variables are filled with the mean, and the categorical variables are filled with the mode. After processing, it is guaranteed that the dataset has no missing values.

*(2) Feature Divergence Analysis*. According to the principles of statistical knowledge and feature selection, the divergence of features is calculated and analyzed; variance is used to measure divergence, and features with a threshold greater than 0.1 are retained.

### 3.2. IV_Cluster Methodology

The IV feature selection method is a supervised feature selection method. It is a filtering feature selection method. By calculating the variable IV value, according to the level of the IV value and the feature selection strategy, it can quickly select Top-K or Top-Percent's feature set. This method has the advantages of a filtered feature selection method, and at the same time, it also has good interpretability.

The IV_Cluster method is an improved feature selection method. On the one hand, it takes advantage of the advantages of clustering, that is, the largest similarity within the class and the largest difference between the classes, and on the other hand, it takes advantage of the advantages of IV, that is, it is efficient and easy to explain. This method first performs unsupervised clustering learning on the variable set to divide some target clusters, then selects the feature with the largest IV value from the target cluster as the representative, and finally combines these representative features to obtain the selected feature set. The IV_Cluster feature selection method can be expressed by the following formula:

(4) $$\begin{array}{c} {\text{Argmax}}_{f_{j}}=IV\left(f_{j}\subset C_{i}\right), \end{array}$$

where *C*_*i*_ is the *i*th variable cluster, *i* = 1, 2..*K* and *f*_*j*_ is the feature set belonging to *C*_*i*._

The calculation of the IV of the variable can be calculated according to the Formula (2), and the method of variable clustering adopts the K-means algorithm [27]. The pseudocode of the IV_Cluster feature selection method, see Algorithm 1:

## 4. Result and Analysis

### 4.1. Metrics

In this paper, we use the 10-fold cross-validation [28] method for the preprocessed dataset using feature selection. Evaluate the Accuracy value [29] and Kappa value [30] of the LR model under different feature sets.

#### 4.1.1. Accuracy

For the binary classification problem, the sample can be categorized into four cases: true positive (TP), false positive (FP), true negative (TN), and false negative (FN), according to the combination of its real category and the classifier prediction category. The TP, FP, TN, and FN represent the corresponding samples. The “confusion matrix” of the classification result is shown in Table 1.

According to the confusion matrix, the accuracy, precision, and recall can be defined. Accuracy is the correct proportion of all predictions and is defined as

(5) $$\begin{array}{c} \text{Accuracy}=\frac{TP+TN}{TP+FP+FN+TN}. \end{array}$$

#### 4.1.2. Kappa

The Kappa value is an indicator used for consistency check, that is, whether the model prediction results are consistent with the actual classification results. For binary classification problems, Kappa is defined as follows:

(6) $$\begin{array}{c} \text{Kappa}=\frac{P_{0}-P_{e}}{1-P_{e}}, \end{array}$$

where *P*_0_ = ∑_*i*=1_^2^*p*_*ii*_ and *P*_*e*_ = ∑_*i*=1_^2^*p*_*i*._*p*_.*i*_

### 4.2. Results

The model evaluation indicators Accuracy and Kappa of P53 under different feature sets 5, 15, and 25 are shown in Table 2.The error bar of Accuracy under the feature set 5, 15, and 25 of the P53 dataset is shown in Figure 1.The error bar of Kappa under the feature set 5, 15, and 25 of the P53 dataset is shown in Figure 2.

Through the results in Table 2 and Figures 1 and 2, we can find that the IV feature selection method of fusion variable clustering proposed in this paper is effective. First of all, for the problem of small sample high-dimensional data, it is necessary to perform the preprocessing operation of feature selection to reduce and eliminate redundant and useless feature sets. Through the experimental results, we found that the P53 protein recognition performance of the former was significantly improved compared with the latter when the feature selection method was used and the feature selection method was not used. Secondly, the IV feature selection method that integrates variable clustering, compared with the filter-type IV feature selection method, the recognition power of P53 is improved in the three sets of feature set tests, and the accuracy rates are increased by 4.4%, 2.0%, and 5.8%, respectively, the Kappa value increased by 21.8%, 8.6%, and 22.4%, respectively. Finally, in order to more robustly compare and analyze the utility of feature selection, we used 10-fold cross-validation, and plotted the error curve for each case, the performance improvement can be intuitively felt by the mean, and the standard error can be a dispersion of properties was observed. Comparing with and without feature selection, we find that the performance of the model is significantly improved and the performance is more robust.

## 5. Discussion

In this paper, we design and propose a new feature selection algorithm for the problems and challenges brought by the actual small sample high-dimensional tumor clinical medical dataset.

In the problem of real small-sample high-dimensional clinical medical data, the number of samples is small, and the number of variables is large, which will lead to the redundancy and similarity of variables. The filtering feature selection algorithm uses a scoring mode to measure the relationship between variables and targets, which is concise and effective, but ignores the relationship and structure between variables. Therefore, on the basis of IV algorithm, we further consider the structure between variables, and design a new feature selection method that integrates variable clustering and IV.

This new algorithm adopts an integration strategy, on the one hand, it absorbs the advantages and interpretability of the information value (IV) feature selection algorithm and, on the other hand, it considers the ability of unsupervised learning to acquire potential internally similar structures.

We tested and verified the P53 proteome dataset of colorectal cancer, and observed the accuracy of the model and the consistency between the model prediction results and the actual results. It was found that the new feature selection algorithm proposed in this paper is effective. Firstly, compared with without the feature selection algorithm, the performance of the model has been significantly improved. This suggests that feature selection is an effective approach in dealing with small sample and high-dimensional problems. Secondly, compared with the information value feature selection algorithm, the performance of the model has been further improved. This shows that integrating feature selection strategy and considering the internal structure of feature sets can help to select more effective feature sets. Thirdly, this new algorithm is helpful for the interpretability of the model. In this paper, we tested three feature sets. These small feature sets are helpful for clinical practitioners in attribution analysis and practice.

However, this new feature selection algorithm has a hyperparameter, that is, the number of feature selection or the number of variable clustering. To solve this problem, on the one hand, we can absorb the prior knowledge of tumor clinicians to determine the interval of hyperparameters; on the other hand, we can consider some methods to find the best hyperparameters, such as grid search method or random search method. In this paper, the differences of model performance under 5, 15, and 25 feature sets were compared and analyzed by using the prior knowledge of clinicians.

## 6. Conclusion

P53 is a proteomic gene with clinical expression and significance for CRC problems. Aiming at the current situation of small samples of high-dimensional data, a variable clustering IV feature selection method proposed in this paper improves the recognition of P53 and has a certain value for clinical guidance of CRC problems. The follow-up research will start from the following two aspects: on the one hand, continue to study the feature selection method for small sample high-dimensional data; on the other hand, consider new model construction methods, such as the design and construction of ensemble models.

## Figures and Tables

**Figure 1:** Accuracy error bar for feature sets. (a) 5 features and all features. (b) 15 features and all features. (c) 25 features and all features.

**Figure 2:** Error bar of Kappa under feature sets. (a) 5 features and all features. (b) 15 features and all features. (c) 25 features and all features.

**Algorithm 1:** Pseudocode of IV_Cluster Methodology.

**Table 1:** Confusion matrix of the classification.

Actual	Predicted positive	Predicted negative
Positive	TP (true positive)	FN (false negative)
Negative	FP (false positive)	TN (true negative)

**Table 2:** Accuracy and Kappa values of the model under different eigenvalues of the P53 dataset are as follows: min, mean, and max.

Metrics	Condition	Feature	Min	Mean	Max
Accuracy	IV_Cluster_LR	5	0.60	**0.67**	0.77
	IV_LR	5	0.57	0.64	0.74
	IV_Cluster_LR	15	0.62	**0.71**	0.86
	IV_LR	15	0.57	0.70	0.83
	IV_Cluster_LR	25	0.57	**0.73**	0.89
	IV_LR	25	0.56	0.69	0.83
	ALL_LR	ALL	0.34	0.49	0.66
Kappa	IV_Cluster_LR	5	0.19	**0.34**	0.54
	IV_LR	5	0.11	0.28	0.48
	IV_Cluster_LR	15	0.23	**0.42**	0.71
	IV_LR	15	0.14	0.38	0.66
	IV_Cluster_LR	25	0.14	**0.45**	0.77
	IV_LR	25	0.10	0.37	0.65
	ALL_LR	ALL	-0.29	-0.01	0.32

## Data Availability

Our data are needed for subsequent studies and are not available at this time.
